The article "Analysis of Sports Injury Estimation Model Based on Mutation Fuzzy Neural Network" was retracted in 2023. Reasons: unreliable results or conclusions; concerns about the data; concerns about the peer review; concerns about the citations.

# Analysis of Sports Injury Estimation Model Based on Mutation Fuzzy Neural Network

**DOI:** 10.1155/2021/3056428

**Published:** 2021-12-01

**Authors:** Dong Wang, Jeng-Sheng Yang

**Affiliations:** ^1^College of Sports Rehabilitation, Shanxi Medical University, Taiyuan, Shanxi 030001, China; ^2^Graduate Institute of Sport Coaching Science, College of Kinesiology and Health, Chinese Culture University, 55, Hwa-Kang Rd, Yang-Mung-Shan, Taipei, Taiwan 11114, China; ^3^Department of Physical Education, Chinese Culture University, 55, Hwa-Kang Rd, Yang-Mung-Shan, Taipei, Taiwan 11114, China

## Abstract

In recent years, with the gradual development of sports, the competition between athletes is becoming more and more fierce. The long training time and heavy body load of athletes lead to the increase of the incidence of sports injury, and the evaluation and analysis of athletes' sports injury need a lot of manpower and material resources. In order to improve the calculation efficiency of sports injury estimation results and save the cost of estimation and analysis, we propose a sports injury estimation model based on the algorithm model of mutation fuzzy neural network. The sports injury model constructed in this paper can not only systematically evaluate and analyze the degree of sports injury of athletes, but also improve the accuracy and efficiency; at the same time, it has universality for the evaluation and analysis of the degree of sports injury. The construction of this model provides the theoretical basis of big data algorithm for the prevention of sports injury and the application of mutation fuzzy neural network in the field of sports.

## 1. Introduction

Artificial neural network (ANN) is an algorithm developed by artificial intelligence imitation on the basis of biological neural system model. With the development of science and technology, it has been widely used in various fields of life [1–3]. The algorithm models of these neural networks are called artificial neural network model, or neural network model [4, 5]. In many neural network models, the development of fuzzy neural network has been concerned [6, 7]. Neural network is generally used to analyze some complex functional relationships between massive data, which involves many steps, including storing knowledge in the weight coefficient and so on. Weight coefficient can be learned from input and output samples, which is characterized by automation and distributed storage [8, 9]. And the neural network algorithm involves a large number of neurons, which makes the whole system run after a large amount of calculation [10, 11]. Fuzzy system has different characteristics. Fuzzy system can summarize and express corresponding knowledge based on human experience, which is more convenient to understand [12–14]. In fuzzy system, knowledge is stored in the rule set, and the number of rules can be controlled and adjusted, which is less than the calculation of neural network [15]. However, rules are mainly provided or designed by experts, which makes the acquisition of rules cost and difficult. Based on their respective advantages and disadvantages, a mutation fuzzy neural network is formed by combining the two. This model will show excellent results in dealing with large-scale data analysis problems and has very good development potential and space [16, 17].

The article "Analysis of Sports Injury Estimation Model Based on Mutation Fuzzy Neural Network" was retracted in 2023. Reasons: unreliable results or conclusions; concerns about the data; concerns about the peer review; concerns about the citations.

Fuzzy neural network (FNN) is based on the fuzzy system and neural network, which combines the two to make up for their disadvantages and give full play to their advantages, improve the efficiency of algorithm operation and the accuracy of output results, and can process fuzzy information [18]. The input and output nodes represent the input and output data signals, respectively, and the implied nodes represent membership functions and fuzzy rules [19]. Fuzzy neural network is based on the further development of fuzzy system model. In the fuzzy neural network algorithm system, each node has a clear physical meaning, and the initial value of these parameters can be determined by the system or qualitative knowledge. On the basis of this step, the learning algorithm is used to quickly analyze and calculate the input-output relationship. The above is the advantage of fuzzy neural network that is different from simple neural network. At the same time, it has neural network structure and is easy to learn and adjust parameters, which is its advantage over simple fuzzy logic system. With the continuous progress of science and technology, now more and more aspects and fields can use the algorithm of combining fuzzy model and neural network to solve practical problems, such as solving some controller structure problems in engineering [20]. In addition, the fuzzy neural network can also be used to solve sports problems, such as the systematic evaluation and analysis of athletes' sports injury degree. In recent years, with the gradual development of the sports field, sports events are becoming more and more fierce, which is accompanied by the competition between athletes. Long training time and heavy body load of athletes lead to an increase in the incidence of sports injury, which seriously affects the maintenance and improvement of athletes' performance, and even leads to athletes' early withdrawal from the competition. The development of artificial intelligence and big data makes the application of algorithm model in this field possible. Therefore, the model development and exploration of sports injury treatment and evaluation through big data have become an important topic in this field.

The article "Analysis of Sports Injury Estimation Model Based on Mutation Fuzzy Neural Network" was retracted in 2023. Reasons: unreliable results or conclusions; concerns about the data; concerns about the peer review; concerns about the citations.

In order to improve the calculation efficiency of sports injury evaluation results and save the cost of evaluation and analysis, a sports injury evaluation model based on mutation fuzzy neural network algorithm model is proposed. The innovative sports injury model constructed in this paper can not only systematically evaluate and analyze the sports injury degree of athletes but also improve the accuracy and efficiency of evaluation. At the same time, the evaluation and analysis of sports injury degree is universal. The establishment of the model provides a theoretical basis for the application of big data algorithm for sports injury prevention and mutation fuzzy neural network in the field of sports.

## 2. Related Work

The development process of fuzzy neural network is very long. Since cybernetics was born in the United States in the 1940s, it has gone through the key development period of classical control theory and modern control theory. However, in the face of some problems with complex data relations, the traditional control theory is still unable to solve well. The existence of these problems urges people to explore more theoretical possibilities. In the early days, there were few researches on the application of fuzzy model to neural network. The first application of fuzzy system combined with neural network dates back to 1974. Subsequently, the development of the theory has not received much in-depth exploration. Wong et al. [21] systematically discussed the possibility of applying fuzzy model to neural network algorithm. Since then, more and more attention has been paid to how to combine the traditional control theory and apply it to neural network to form intelligent control theory.

With the continuous development of science and technology, the algorithm model formed by the combination of fuzzy system and neural network has been widely used in many fields. Kuo and Zulvia [22] applied gradient evolution algorithm to an intuitionistic fuzzy neural network for forecasting medical cost. Next, Yang et al. [23] proved that fuzzy systems with product reasoning, central antifuzzification, and Gaussian membership functions can also approximate real continuous functions on any closed subset with any precision. Introducing fuzzy control technology into the learning algorithm can dynamically adjust the learning process of the network and make the traditional static learning algorithm dynamic, such as the fuzzy logic control technology of backward propagation algorithm of layered perceptron given by Baskin et al. [24]. In recent years, many domestic scholars have studied the training algorithm of neural network, mainly focusing on the rapidity of neural network training, global optimization technology, and generalization ability [25].

The article "Analysis of Sports Injury Estimation Model Based on Mutation Fuzzy Neural Network" was retracted in 2023. Reasons: unreliable results or conclusions; concerns about the data; concerns about the peer review; concerns about the citations.

To sum up, with the development of science and technology, the combined application of fuzzy network and neural network has better development potential and larger expansion space. This paper introduces the development process and basic principle of fuzzy network and neural network. In addition, based on the advantages of this algorithm, this paper proposes a sports injury estimation model applied to a variety of sports fields.

## 3. Construction of Sports Injury Estimation Model Based on Fuzzy Neural Network

### 3.1. Construction of Fuzzy Neural Network

Fuzzy theory and neural network technology are two active fields of artificial intelligence research in recent years. Artificial neural network is a thinking function simulating the structure of human brain. It has strong self-learning and association functions, less manual intervention, high precision, and better utilization of expert knowledge. Fuzzy logic is an extension of ordinary binary logic, which truly reflects all statements, and its value range is real numbers between 0 and 1. The fuzzy set used in fuzzy neural network can be expressed by the following formula.

The union is expressed as

(1) $$\begin{array}{c} \mu_{A\cup B}\left(x\right)=\mu_{A}\left(x\right)\cup \mu_{B}\left(x\right)=\text{max}\left(\mu_{A}\left(x\right),\mu_{B}\left(x\right)\right). \end{array}$$

The intersection is expressed as

(2) $$\begin{array}{c} \mu_{A\cap B}\left(x\right)=\mu_{A}\left(x\right)\cap \mu_{B}\left(x\right)=\text{min}\left(\mu_{A}\left(x\right),\mu_{B}\left(x\right)\right). \end{array}$$

The complement is expressed as

(3) $$\begin{array}{c} \mu_{A}\neg =1-\mu_{A}\left(x\right). \end{array}$$

The algebraic product is expressed as

(4) $$\begin{array}{c} \mu_{A\cdot B}\left(x\right)=\mu_{A}\left(x\right)\times \mu_{B}\left(x\right). \end{array}$$

The algebraic sum is expressed as

(5) $$\begin{array}{c} \mu_{A+B}\left(x\right)=\mu_{A}\left(x\right)+\mu_{B}\left(x\right)-\mu_{A}\left(x\right)\cdot \mu_{B}\left(x\right). \end{array}$$

The Gauss membership function is expressed as

(6) $$\begin{array}{c} \mu \left(x\right)=\text{exp}\left(-\frac{{\left(x-c\right)}^{2}}{\sigma^{2}}\right). \end{array}$$

Fuzzy system is a dynamic model with fuzzy information processing ability based on fuzzy rules. In fuzzy system, there are four basic parts, and the diagram is shown in Figure 1. As can be seen from Figure 2, the four basic parts are fuzzifying interface, knowledge base, fuzzy inference engine, and the final antifuzzifying interface [26, 27].

The article "Analysis of Sports Injury Estimation Model Based on Mutation Fuzzy Neural Network" was retracted in 2023. Reasons: unreliable results or conclusions; concerns about the data; concerns about the peer review; concerns about the citations.

The same as fuzzy logic, neural network is also a very important control algorithm, both through different research angles to explore the problem of understanding. On the one hand, the fuzzy system solves the problem of fuzziness by imitating the neural thinking of the brain from the macro point of view; on the other hand, the neural network starts from the micro point of view, starting from the simulation of neurons, learning and parallel processing massive data on the basis of imitating the function of organisms. There is a certain connection between the two, which can maximize the advantages and make up for the disadvantages [28, 29].

In the fuzzy neural network algorithm, similar to PID algorithm, multilayer feedforward neural network is a feedback algorithm, which has better accuracy and optimization ability.  Figure 3 shows the structure model of fuzzy neural network. The back-end network is used to generate fuzzy rules, and the front-end network is used to match the generated fuzzy rules with each layer [30].

In FNN, there are five layers: input layer, fuzzification layer, fuzzy rule antecedent matching layer, fuzzy rule antecedent matching layer, and defuzzification layer. The calculation formula involved in each layer is as follows.

In the input layer, each input data are the index data of sports injury degree, and each node is a component of the input sample, which is expressed as

(7) $$\begin{array}{c} O_{i}^{l}=I_{i}^{l},\;i=1,2,3. \end{array}$$

In the fuzzification layer, the output value of the node is the membership value, which is expressed by Gaussian function [31–34].

(8) $$\begin{array}{c} I_{j}^{2}=O_{j}^{l},\\ O_{j}^{2}=f\left(I_{j}^{2}\right)=\text{exp}{\left(-\frac{I_{j}^{2}-m_{t}}{\delta_{t}}\right)}^{2}, \end{array}$$

where *m*_*t*_ and *δ*_*t*_ represent the center and width of the membership function.  *j*, *t*=1,2,…, 8.

In the antecedent matching layer of fuzzy rules, nodes are responsible for performing operations.

(9) $$\begin{array}{c} I_{k}^{3}=\prod_{j}O_{jk}^{2}=O_{k}^{3}. \end{array}$$

In the fuzzy rule consequent matching layer, the nodes need to input and calculate the consequent of the same rule in the process of operation.

(10) $$\begin{array}{c} I_{l}^{4}=\sum_{k}\omega_{kl}^{4}O_{k}^{3}. \end{array}$$

In which,

(11) $$\begin{array}{c} O_{l}^{4}=\text{min}\left(1,I_{l}^{4}\right), \end{array}$$

*ω*_*kl*_^4^ is the rule weight, where *l*=1,2,3.

In the defuzzification layer, the principle of maximum membership degree is adopted

(12) $$\begin{array}{c} I^{5}=O_{l}^{4},\\ u=\text{max}\left(I_{1}^{5},I_{2}^{5},I_{3}^{5}\right). \end{array}$$

The second and third layer nodes of fuzzy neural network will increase exponentially with the increase of input variable data, and the third layer also changes exponentially. When the amount of input data and output data increase sharply in the network, a series of related values such as the number of nodes and the weight of output will also change rapidly and increase sharply. Therefore, this kind of network has high requirements for the forward calculation of the system and the reverse transmission on the network. In some cases, it will affect the operation speed to a certain extent.

The article "Analysis of Sports Injury Estimation Model Based on Mutation Fuzzy Neural Network" was retracted in 2023. Reasons: unreliable results or conclusions; concerns about the data; concerns about the peer review; concerns about the citations.

As a combination of fuzzy system and neural network algorithm, fuzzy neural network not only has the advantages of both but also makes up for the defects of both. In this paper, the sports injury degree estimation model based on mutation fuzzy neural network has the advantages of high accuracy and efficiency, which provides a reference for the application of the model in more fields in the future.

### 3.2. Construction of Sports Injury Estimation Model

Sports injury is caused by sports. Athlete's injury refers to all kinds of injuries related to football training and competition, which hinder the athlete's movement or require special treatment (such as special bandage and medical treatment) in order to continue the movement, or this kind of injury completely prevents the athlete's movement. There is no unified standard to judge sports injury. It is generally believed that the athletes cannot participate in training and competition and need medical treatment and diagnosis of organic tissue injury.

In the process of evaluating the degree of sports injury, the most important step is to determine the relevant fuzzy set. Assuming that the corresponding damage degree level is a fixed value, the damage degree index is quantified through the process of fuzzy set index quantification. After quantification, these damage-related indicators can be divided into five categories, including damage location, damage link, and other influencing factors. For the evaluation and analysis indicators of the degree of injury, this paper is divided into three evaluation indicators, mainly related to the degree of physical health, the difficulty of injury recovery, and the impact of mental state. The classification is shown in Figure 4.

On the basis of mutation fuzzy neural network algorithm, we use *d*_*j*_ to express the three evaluation indexes, where *j* = 1,2,3. The degree of damage is set to *x*_*j*_, and the number of damage is set to *k.* Therefore, after *k* times of damage, the evaluation result can be expressed as *k.*, where *j* = 1,2,3, and the membership degree *r*_*j*_ can be expressed as

(13) $$\begin{array}{c} r_{j}=\frac{E_{j}}{k}. \end{array}$$

After calculation, the value of damage fuzzy set can be expressed as

(14) $$\begin{array}{c} D=\sum_{j=1}^{3}\left(r_{j}\times x_{j}\right). \end{array}$$

In the process of evaluating and analyzing the damage degree of the damaged part, we need to determine three groups of weight values, including the influencing factors of the damaged part, the damage mode, and the required recovery ability after the damage, which can be expressed by the following formula.

The article "Analysis of Sports Injury Estimation Model Based on Mutation Fuzzy Neural Network" was retracted in 2023. Reasons: unreliable results or conclusions; concerns about the data; concerns about the peer review; concerns about the citations.

The influencing factors of injury site were as follows:

(15) $$\begin{array}{c} Z=\left\{z_{1},z_{2},\ldots ,z_{9}\right\}. \end{array}$$

The damage mode can be expressed as

(16) $$\begin{array}{c} E=\left[\begin{array}{c} \begin{array}{ccc} e_{11} & e_{12} & \begin{array}{cc} \cdots & e_{19} \end{array}\\ e_{21} & e_{22} & \begin{array}{cc} \cdots & e_{29} \end{array}\\ \vdots & \vdots & \begin{array}{cc} \ddots & \vdots \end{array} \end{array}\\ \begin{array}{ccc} e_{91} & e_{92} & \begin{array}{cc} \cdots & e_{99} \end{array} \end{array} \end{array}\right]. \end{array}$$

The damage influence matrix *E* is used as the test formula of the model to ensure the influence of different damage modes on the evaluation accuracy to a certain extent.

The ability to recover from injury can be expressed as

(17) $$\begin{array}{c} \left\{\begin{array}{c} ife_{hk}>e_{hl},\;{\text{thene}}_{lk}>e_{kl},\\ ife_{hk}<e_{hl},\;{\text{thene}}_{lk}<e_{kl},\\ ife_{hk}=e_{hl},\;{\text{thene}}_{lk}=e_{kl}. \end{array}\right) \end{array}$$

Among them, *e*_*hk*_ is the average recovery ability; *e*_*hl*_ was the average recovery ability of sports injury; *e*_*lk*_ is the external restoration aid; and *e*_*kl*_ is the best external auxiliary ability. Through the internal and external comparison, the influence of the ability of injury recovery on the evaluation results of sports injury degree can be seen directly through the formula.

For the integrity of the design, we need to verify the final evaluation results of the analysis, and we need to use the weight equation in the process of verification. One of the advantages of weight equation is that it can be used in vector computation. Vector calculation can measure the direction of an estimated value and evaluate the result. The calculation formula is as follows:

(18) $$\begin{array}{c} C=W_{s}\times D+W_{P}\times P, \end{array}$$

where *C* is the vector value of damage degree evaluation analysis results; *D* is the vector value of influencing factors of damage location; *P* is the quantitative value of damage degree; and *W*_*s*_ and *W*_*P*_ are used to express the weight and formal weight of the damage recovery ability.

The article "Analysis of Sports Injury Estimation Model Based on Mutation Fuzzy Neural Network" was retracted in 2023. Reasons: unreliable results or conclusions; concerns about the data; concerns about the peer review; concerns about the citations.

The schematic diagram of the sports injury estimation model is as follows.

As shown in Figure 5, in the sports injury treatment model constructed in this paper, we quantify the specific situation of sports injury according to the three evaluation indexes set above and get the initial sample data, which mainly includes the index values of three modules: physical health degree, injury recovery difficulty, and mental state. Then, the quantitative data are input as the input sample of the fuzzy neural network, and the comprehensive evaluation and analysis results of the degree of sports injury are obtained through the mutation fuzzy neural network algorithm.

### 3.3. Sports Injury Estimation Model Based on Mutation Fuzzy Neural Network

We combine the sports injury model with the fuzzy neural network. While constructing the evaluation model based on the mutation fuzzy neural network, we also explain the divergence of the statistical data, that is, the data mutation index. Mutation index is a very important index, which can help us understand the overall characteristics of data. The mutation index plays an important role in outlier detection. In this paper, the mutation index is used to improve the fuzzy neural network algorithm, and the improved algorithm is suitable for multidimensional numerical data.

In the evaluation model of sports injury, the determination of characteristic membership function and fuzzy inference rules is actually a problem of finding the optimal parameters in the parameter space. Compared with other algorithms, genetic algorithm has better robustness and global, so it has better optimization effect for neural network, fuzzy system, and other algorithms dealing with massive complex data and can greatly improve the accuracy and efficiency of the original algorithm. In this paper, on the basis of fuzzy neural network algorithm, genetic algorithm is used to optimize it, including the optimization of membership function parameters and rule weights, so as to expand the advantages of the combination of the algorithm and obtain more accurate and reliable results in the evaluation and analysis of the degree of sports injury. The specific process is shown in Figure 6.

In this study, the genetic algorithm is used to optimize the fuzzy neural network, and on this basis, the membership function parameters and rule weight values are optimized, so as to obtain a simplified, stable, and reliable algorithm model.

## 4. Experimental Results and Analysis

After the construction of the sports injury estimation model based on the mutation fuzzy neural network, this paper analyzes through experiments and takes the Bayesian model and Lagrange Model as the comparison model of sports injury estimation, so as to carry out the estimation analysis of accuracy and efficiency. As shown in Figure 7, the comparison results of the accuracy of three different models in the estimation and analysis of sports injury results are shown.

The article "Analysis of Sports Injury Estimation Model Based on Mutation Fuzzy Neural Network" was retracted in 2023. Reasons: unreliable results or conclusions; concerns about the data; concerns about the peer review; concerns about the citations.

As can be seen from Figure 7, the accuracy of Bayesian model and Lagrange Model for the estimation of sports injury starts to maintain at about 80%, but with the increasing sample size, the accuracy of the evaluation also gradually decreases. When the sample size reaches 50, the evaluation accuracy of the two comparative models drops to about 60%. The results of the evaluation and analysis of the sports injury degree by the model of the mutation fuzzy neural network show that the model of the mutation fuzzy neural network keeps a high precision level in the whole process of increasing the sample size from 10 to 50, and the precision is more than 90%. The results show that the model constructed in this paper gives full play to the advantages of fuzzy system and neural network algorithm in accuracy level and has obvious improvement in accuracy.

In addition, we also make a comparative analysis of the evaluation efficiency of the three models. The comparison results of three different models are shown in Figure 8.

It can be seen from the comparison results in Figure 8 that with the increasing number of samples processed by abscissa analysis, the time curve of the mutation fuzzy neural network model constructed in this paper is always lower than that of Bayesian model and Lagrange Model, indicating that its operation efficiency is higher than that of the two comparison models. The model in this paper can maintain the same high efficiency, which fully reflects the advantages of fuzzy neural network.

In order to test the difference between the evaluation results of the model constructed in this paper and other models, based on the sports injury estimation model of the mutation fuzzy neural network, we set the injury model with the same index, and then add another two models, namely Bayesian model and Lagrange Model, for unified evaluation and analysis. The results are shown in Figure 9.

It can be seen from Figure 9 that for the same degree of sports injury, the evaluation results of the three models are different to a certain extent, mainly due to the differences in the analysis accuracy of the three models shown. For the agreed degree of injury, higher accuracy can make the analysis results more accurate and reliable, while processing a large number of samples, it can maintain a good judgment index standard and reduce unnecessary errors, which plays an important role in the application of mutation fuzzy neural network algorithm to the parameter evaluation of more sports fields, including sports injury degree evaluation and analysis. It provides a reliable theoretical basis for the extension of the mutated fuzzy neural network in the field of sports.

The article "Analysis of Sports Injury Estimation Model Based on Mutation Fuzzy Neural Network" was retracted in 2023. Reasons: unreliable results or conclusions; concerns about the data; concerns about the peer review; concerns about the citations.

In addition, we also take the common sports injuries of football players as an example to test the analysis results of the sports injury degree estimation analysis model based on the mutation fuzzy neural network. Football is one of the most popular sports in the world. In its sports events and ordinary training, athletes' sports injury accidents often occur, and the probability is about 10–35 cases per 1000 hours. At the same time, the degree of injury is also positively related to the intensity of the game. Therefore, it will be an important work to estimate and analyze the degree of injury of football players. Through big data and artificial neural network algorithm, a lot of human resource costs can be saved. As shown in Figure 10, the algorithm model constructed in this paper analyzes the experimental results of the samples of football injury in China.

First of all, we divide the injury degree of football players into five degrees, namely, A, B, C, D and E, according to the index given by experts, which represent the five degrees of micro, light, medium, high, and dangerous in turn. Then we mix all the samples and input the samples into the algorithm model constructed in this paper for experimental testing and get the evaluation results of these five degrees of damage. From the analysis results in Figure 9, it can be seen that the sports injury degree estimation model based on the mutation fuzzy neural network algorithm constructed in this paper has good recognition ability, and its evaluation and analysis ability have little difference from the index of manual analysis, which ensures good accuracy, and indicates the reliability of the algorithm to a certain extent. It provides a good theoretical basis for the algorithm to replace manual analysis in the future.

Next, we also use the model constructed in this paper to analyze the damage degree of different sports and make the error comparison, and the results are shown in Figure 11.

The results show that for different sports, the model constructed in this paper has high accuracy, and the error value is not more than 1. Among the various sports tested, the accuracy of the results of sports injury estimation and analysis related to riding and football need to be improved, while the accuracy of sliding sports has a very low error value, which is quite high. Through this experiment, it can be proved that the model constructed in this paper can be widely used in various sports, including but not limited to the sports tested in this paper, which shows that the model has excellent performance in the estimation and analysis of sports injury degree of various sports, and shows that the model has good universality and high accuracy.

The article "Analysis of Sports Injury Estimation Model Based on Mutation Fuzzy Neural Network" was retracted in 2023. Reasons: unreliable results or conclusions; concerns about the data; concerns about the peer review; concerns about the citations.

## 5. Conclusion

Based on the algorithm model of mutation fuzzy neural network, this paper proposes and constructs a sports injury estimation and analysis model for athletes. Through the combination of fuzzy model and neural network algorithm, we can make up for their disadvantages and give full play to their advantages, so as to improve the efficiency of the algorithm and the accuracy of the output results. Through the experimental verification, compared with Bayesian model and Lagrange Model, the sports injury estimation model based on the mutation fuzzy neural network constructed in this paper has higher accuracy and efficiency. For the same kind of sports injury, the results of this model are close to the results of artificial evaluation and analysis to a certain extent, which can greatly improve the operation efficiency and have certain data reliability at the same time. For different sports, the model has a low degree of error, which indicates that it is universal for the estimation and analysis of the degree of injury in various sports. The sports injury estimation model based on the mutation fuzzy neural network constructed in this study can systematically evaluate and analyze the sports injury degree of athletes and provide the theoretical basis of big data algorithm for preventing sports injury and ensuring the safety of athletes. However, the algorithm model proposed in this paper is the result of computer simulation and manual evaluation. There is still a certain gap between the practical application and the reality, and the research data need to be further expanded for verification in the future research work.

## Figures and Tables

**Figure 1:** The constitution of fuzzy systems.

**Figure 2:** Photo of measuring sensor.

**Figure 3:** The structure of fuzzy neural network.

**Figure 4:** Sports injury risk factors and injury degree indexes.

**Figure 5:** Schematic diagram of sports injury estimation model.

**Figure 6:** Flowchart of sports injury estimation model based on mutation fuzzy neural network.

**Figure 7:** Comparison results of the accuracy of sports injury estimation of the three models: the mutation fuzzy neural network model, the Bayesian model, and the Lagrange model.

**Figure 8:** Comparison results of the evaluation efficiency of the three models, namely, the mutation fuzzy neural network model, the Bayesian model, and the Lagrange model.

The article "Analysis of Sports Injury Estimation Model Based on Mutation Fuzzy Neural Network" was retracted in 2023. Reasons: unreliable results or conclusions; concerns about the data; concerns about the peer review; concerns about the citations.

**Figure 9:** Comparison results of different models for the same damage degree.

**Figure 10:** Analysis results of different degree of injury in football.

**Figure 11:** Accuracy comparison chart of injury degree assessment in different sports.

## Data Availability

The data used to support the findings of this study are available from the corresponding author upon request.
